# A Nomogram for Predicting the Mortality of Patients with Acute Respiratory Distress Syndrome

**DOI:** 10.1155/2022/5940900

**Published:** 2022-04-07

**Authors:** Zhenqing Wang, Lihua Xing, Hongwei Cui, Guowei Fu, Hui Zhao, Mingjun Huang, Yangchao Zhao, Jing Xu

**Affiliations:** ^1^Department of Cardiovascular Surgery, The First Affiliated Hospital of Zhengzhou University, Zhengzhou, China; ^2^Department of Respiratory ICU, The First Affiliated Hospital of Zhengzhou University, Zhengzhou, China; ^3^Department of General ICU, The First Affiliated Hospital of Zhengzhou University, Zhengzhou, China

## Abstract

Acute respiratory distress syndrome (ARDS) is an acute lung injury associated with high morbidity and mortality. This study aimed to establish an accurate prediction model for mortality risk in ARDS. 70% of patients from the Medical Information Mart for Intensive Care Database (MIMIC-III) were selected as the training group, and the remaining 30% as the testing group. Patients from a Chinese hospital were used for external validation. Univariate and multivariate regressions were used to screen the independent predictors. The receiver operating characteristic curve (ROC) analysis, the Hosmer–Lemeshow test, and the calibration curve were used for evaluating the performance of the model. Age, hemoglobin, heart failure, renal failure, Simplified Acute Physiology Score II (SAPS II), immune function impairment, total bilirubin (TBIL), and PaO_2_/FiO_2_ were identified as independent predictors. The algorithm of the prediction model was: ln (Pr/(1 + Pr)) = −3.147 + 0.037 ∗ age − 0.068 ∗ hemoglobin + 0.522 ∗ heart failure (yes) + 0.487 ∗ renal failure (yes) + 0.029 ∗ SAPS II + 0.697 ∗ immune function impairment (yes) + 0.280 ∗ TBIL (abnormal) − 0.006 ∗ PaO_2_/FiO_2_ (Pr represents the probability of death occurring). The AUC of the model was 0.791 (0.766–0.816), and the internal and the external validations both confirmed the good performance of the model. A nomogram for predicting the risk of death in ARDS patients was developed and validated. It may help clinicians early identify ARDS patients with high risk of death and thereby help reduce the mortality and improve the survival of ARDS.

## 1. Introduction

Acute respiratory distress syndrome (ARDS) is an acute lung injury characterized by progressive hypoxemia and respiratory distress and is associated with high morbidity and mortality [1–3]. In China, the incidence of ARDS was 27% in the ICU, and the mortality rate was as high as 25% to 75% [4]. The incidence is about 10.4% with the overall incidence of postoperative ARDS of about 3% [5]. Herein, it is of great significance to early identify ARDS patients with higher risk of death and to perform early intervention and treatment, which would help reduce the mortality risk of ARDS and improve the poor prognosis.

At present, many studies have extensively studied the risk factors for mortality of ARDS, including age [6–8], lower respiratory tract infection [8], immunosuppressive drugs [9, 10], multiple organ failures [8, 11], and some biomarkers [12, 13]. However, due to multiple factors that worked together to determine the final outcome of ARDS patients, developing an effective prediction model would be of great clinical use for risk assessment. Currently, most of the established prediction models were limited by the small sample size, single study population, or lacking external validation [14, 15]. Therefore, this study aims to establish an accurate prediction model for mortality risk in ARDS based on the Medical Information Mart for Intensive Care Database (MIMIC-III) and perform external validation in a Chinese population.

## 2. Methods

### 2.1. Study Population

In the retrospective study, we collected patient data from the Medical Information Mart for Intensive Care Database III version 1.3 (MIMIC-III v1.3) for the development of the prediction model. Inclusion criteria were as follows: (1) patients whose age ≥18 years and (2) patients who were diagnosed with ARDS according to the Berlin definition [1]. The MIMIC-III Database is a large, freely accessible database comprising information related to patients admitted to critical care unit at a large tertiary care hospital. It integrates deidentified, comprehensive clinical data of patients admitted to the Beth Israel Deaconess Medical Center in Boston, Massachusetts, and makes it widely accessible to researchers internationally under a data use agreement.

Also, ARDS patients in the First Affiliated Hospital of Zhengzhou University from June 2014 to December 2020 were enrolled in the study for external validation. Inclusion criteria were as follows: (1) patients whose age ≥18 years and (2) patients who were diagnosed with ARDS according to the Berlin definition [1]. The Ethics Committee of the First Affiliated Hospital of Zhengzhou University suggests that retrospective studies be exempted from ethical review. As the present study was a retrospective study, the Ethics Committee of the First Affiliated Hospital of Zhengzhou University exempted it from the requirement of the ethical review. All identifiable information about the patients has been stripped; the Ethics Committee of the First Affiliated Hospital of Zhengzhou University has waived the requirement for the informed consent in the study. Also, the study was conducted in line with the Declaration of Helsinki.

### 2.2. Data Extraction

In the present study, demographic data, laboratory indicators, and clinical data were collected. The following variables were extracted: age (years), sex, SaO_2_, PaO_2_/FiO_2_, platelet (PLT, 109/L), pH, lactate (mmol/L), international normalized ratio (INR, %), creatinine (mg/dl), hematocrit (%), hemoglobin (g/dl), aspartate transaminase (AST, U/L), alanine transaminase (ALT, U/L), total bilirubin (TBIL, umol/L), blood urea nitrogen (BUN, mg/dl), white blood cell (WBC, 109/L), potassium (mmol/L), sodium (mmol/L), bicarbonate (mmol/L), mean arterial pressure (MAP, mm Hg), ICU type, causes of ARDS, bicarbonate input, ventilation, ventilation time, the Simplified Acute Physiology Score II (SAPS II), the Glasgow Coma Scale (GCS), the Sequential Organ Failure Assessment (SOFA) score, immune function impairment, heart failure, renal failure, respiratory rate (breaths/min), and heart rate (breaths/min). Immune function impairment was defined as patients with liver cirrhosis, acquired immune deficiency syndrome (AIDS), solid tumor, hematological malignancy, solid organ transplantation, or long-term use of corticosteroids. Multiple imputation was used to deal with missing data and sensitivity analysis was performed to evaluate the impact on the study after imputation (Table 1).

### 2.3. Development and Validation of the Prediction Model

Firstly, the 70% of the study patients from the MIMIC-III Database were randomly selected as the training group for the development of the prediction model, and the remaining 30% as the testing group for the internal validation. Data of patients from the hospital were used for external validation. After developing the prediction model, we adopted the receiver operating characteristic curve (ROC) analysis, the Hosmer–Lemeshow test, and the calibration curve to evaluate the performance of the model.

Univariate regression analysis was performed using the data of the training group from the MIMIC-III Database. Variables with statistical significance in the univariate analysis were included in the multivariate regression for stepwise screening, to screen the independent predictors and thereby to develop the model. The algorithm of the prediction model is as follows: the dependent variable *y* is 0 (represents survival) and 1 (represents death); the Pr value is the probability of death event.

(1) $$\begin{array}{c} \mathrm{Pr}\left(y=1\right)=\frac{e^{z}}{1+e^{z}}, \end{array}$$

where (*z*=*β*_0_+*β*_1_*∗x*_1_+⋯+*β*_*m*_*∗x*_*m*_).

Then we used the maximum likelihood estimation (MLE) to estimate the coefficients of each variable.

Finally, ln(Pr/1 − Pr)=*β*_0_+*β*_1_*∗x*_1_+⋯+*β*_*m*_*∗x*_*m*_.

### 2.4. Statistical Analysis

Normally distributed measurement data were described as mean ± standard deviation (Mean ± SD), and the independent *t*-test was used for comparison between groups. Nonnormally distributed data were described as median and interquartile range *M* (Q1, Q3), and the Mann-Whitney *U* test was used for comparison. Besides, enumeration data were described as number of cases and constituent ratio *N* (%), and the chi-squared test or Fisher's exact test was used for comparison.

We adopted the univariate and multivariate regression analysis to screen some independent predictors, and thereby these predictors were included in the prediction model to establish a prediction equation for assessing the risk of death in ARDS patients.

For visualizing the prediction model, we also plotted a nomogram. Then, the established model performed the internal and external validation, to assess the predicting performance of model. The receiver operating characteristic curve (ROC) analysis, the Hosmer–Lemeshow test, and the calibration curve were used for evaluating the performance of the model. The two-tailed test was carried out for all statistical tests, and *P* < 0.05 was considered statistically significant. The SAS 9.4 software (SAS Institute Inc., Cary, NC, USA) was used for the screening of independent predictors and the development of the prediction model. R 4.0.2 was used to validate and visualize the model.

## 3. Results

### 3.1. Baseline Description

In the present study, 1,814 patients were randomly selected from the MIMIC-III Database with 1,230 in the training group and 584 in the testing group. The mean age was 62.16 ± 16.93 years. There were 1,048 (57.77%) males and 766 (42.23%) females. The ARDS of 150 (8.27%) patients was caused by pneumonia, the ARDS of 51 (2.81%) was by sepsis, and the ARDS of the remaining 1,613 (88.92%) was by other causes. Impaired immune function was reported in 544 (29.99%) patients, heart failure in 553 (30.49%) patients, and renal failure in 611 (33.69%) patients. 1,550 (85.45%) patients received ventilation and 264 (14.55%) did not, and the median ventilation time was 7.00 (3.00, 15.00) days. The median SAPS II was 38.00 (29.00, 48.00). The median GCS score was 9.00 (5.00, 14.00). The median SOFA score was 6.00 (4.00, 9.00). As shown in Table 2, there were no significant differences in baseline information and laboratory indicators between the randomly selected training group and the testing group (all *P* > 0.05).

In the Chinese hospital, totally 168 eligible patients were included: 100 (59.52%) males and 68 (40.48%) females. The mean age was 61.43 ± 17.66 years.

The ARDS of 7 (4.17%) patients was caused by pneumonia, the ARDS of 2 (1.19%) was by sepsis, and the ARDS of the remaining 159 (94.64%) was by other causes. Among them, 41 (24.40%) patients reported immune function impairment, 52 (30.95%) reported heart failure, and 55 (32.74%) reported renal failure. 21 (12.5%) patients received ventilation and 147 (87.50%) did not, and the median ventilation time was 7.00 (2.50, 14.00) days. The median SAPS II was 36.00 (29.00, 47.00). The median GCS score was 9.00 (5.00, 13.00). The median SOFA score was 6.00 (4.00, 9.00) (Table 2).

### 3.2. Development of the Prediction Model

According to the clinical outcome, the training group was divided into the survival group (*n* = 628) and the death group (*n* = 602). As shown in Table 3, the univariate logistic regression analysis suggested that age (*t* = −14.790, *P* < 0.001), the constituent ratios of immune function impairment (*χ*^2^ = 30.088, *P* < 0.001), heart failure (*χ*^2^ = 69.255, *P* < 0.001), renal failure (*χ*^2^ = 76.323, *P* < 0.001), INR (*Z* = 6.092, *P* < 0.001), creatinine (*Z* = 5.050, *P* < 0.001), abnormal TBIL (*χ*^2^ = 14.059, *P* < 0.001), input bicarbonate (*χ*^2^ = 9.770, *P*=0.002), SAPS II (*Z* = 13.604, *P* < 0.001), and SOFA score (*Z* = 6.820, *P* < 0.001) in the death group were all significantly higher than those in the survival group. The constituent ratios of hematocrit (*t* = 3.440, *P* < 0.001), hemoglobin (*t* = 4.470, *P* < 0.001), abnormal BUN (*χ*^2^ = 26.937, *P* < 0.001), ventilation (*χ*^2^ = 33.480, *P* < 0.001), MAP (*t* = 2.720, *P* = 0.007), and PaO_2_/FiO_2_ (*Z* = −5.321, *P* < 0.001) were all significantly lower than those in the survival group.

Variables with statistical significance in the univariate analysis and the factors in the literature that have an impact on the prognosis of ARDS patients (ARDS causes and ventilation time [16]) were further included in the multivariate logistic regression. As shown in Table 4, the results showed that age, hemoglobin, heart failure, renal failure, SAPS II, immune function impairment, TBIL, and PaO_2_/FiO_2_ were identified as independent predictors of death in ARDS patients. For every one-year increase in age, the mortality risk in ARDS patients increased by 0.037 times (OR = 1.037, 95% CI: 1.028–1.047). For every 1 g/dl increase in hemoglobin, the mortality risk was reduced by 0.066 times (OR = 0.934, 95% CI: 0.877–0.995). The mortality risk of patients with heart failure increased by 0.686 times (OR = 1.686, 95% CI: 1.258–2.258), and the risk increased by 0.628 times (OR = 1.628, 95% CI: 1.217–2.178) for those with renal failure. For every one-point increase in SAPS II, the mortality risk increased by 0.029 times (OR = 1.029, 95% CI: 1.020–1.039). The risk increased by 1.007 times (OR = 2.007, 95% CI: 1.498–2.689) in patients with immune function impairment and 0.322 times (OR = 1.322, 95% CI: 1.013–1.727) in those with abnormal TBIL. For every unit increase in PaO_2_/FiO_2_, the risk was reduced by 0.005 times (OR = 0.995, 95% CI: 0.990–0.999).

Then we used the MLE to estimate the coefficients of each variable, and the algorithm of the prediction model was as follows: ln (Pr/(1 + Pr)) = −3.147 + 0.037 ∗ age − 0.068 ∗ hemoglobin + 0.522 ∗ heart failure (yes) + 0.487 ∗ renal failure (yes) + 0.029 ∗ SAPS II + 0.697 ∗ immune function impairment (yes) + 0.280 ∗ TBIL (abnormal) − 0.006 ∗ PaO_2_/FiO_2_ (Pr represents the probability of death occurring). For visualizing the prediction model, we also plotted a nomogram (Figure 1). For example, as shown in Figure 2, the patient was 67.2 years old with normal TBIL. The hemoglobin was 7.4 g/dL and PaO_2_/FiO_2_ was 22.2. SAPS II was 38. The patient was complicated with renal failure and immune function impairment, but no heart failure was reported. According to the nomogram, the total number of points was 373 and the corresponding predicted probability was 0.728, which indicated a high risk of death and was in line with the actual outcome of the patient.

### 3.3. Assessment and Validation of the Prediction Model

According to the ROC analysis, the AUC value of the training group was 0.791 (0.766–0.816), and the AUC was 0.780 (0.743–0.816) in the testing group (Table 5), all suggesting the good discrimination of the model. The Hosmer–Lemeshow test (*χ*^2^ = 49.123, *P* = 0.107), the ROC curves, and the calibration curves all indicated the good discrimination and calibration of the model (Figure 3). The Youden index suggested the cutoff value of 0.458. In the external validation, the AUC was 0.758 (0.756–0.761) (Table 5). The Hosmer–Lemeshow test (*χ*^2^ = 7.256, *P* = 0.509) and the calibration curves both suggested the good performance of the model in Chinese patients (Figure 3).

## 4. Discussion

In the present study, the prediction model based on eight predictors, age, heart failure, renal failure, immune function impairment, hemoglobin, TBIL, PaO_2_/FiO_2_, and SAPS II, was developed with good discrimination and calibration. The internal validation and external validation both confirmed the good performance of the model as reflected by the ROC analysis, the Hosmer–Lemeshow test, and the calibration curve. This may help clinicians predict the individual risk of death in ARDS patients.

Respiratory system dysfunction is often characterized by hypoxemia and impairment of gas exchange with the most developed form as ARDS [17, 18]. In the model, with the increase of hemoglobin and the oxygenation index of PaO_2_/FiO_2_, the risk of death was decreased. Villar et al. reported similar findings that patients with more severe lung disease tend to have lower PaO_2_/FiO_2_ [15]. Our model also found that an older age was associated with an increased risk of death in ARDS patients. This was consistent with previous studies [6, 7, 12]. The body may experience functional degeneration such as immune function impairment with the increase of age, leading to the decline of respiratory capacity and antibacterial capacity. In addition, older patients with ARDS may be complicated by other systemic diseases. The results of this study showed that both heart failure and renal failure independently increased the risk of death from ARDS. This was consistent with previous findings that multiple organ failures were responsible for death in ARDS patients [18, 19]. Moran et al. found that although the proportion of severe ARDS patients who died of respiratory failure alone decreased, the number of deaths from multiple organ failures increased year by year [20]. Herein, in clinical treatment, attention should be paid not only to the elderly patients but also to the deterioration of ARDS caused by other systemic failures.

To our knowledge, there are few studies that have established prediction models for assessing the risk of death in ARDS patients [14, 15, 21]. The model developed by Gajic O et al. was well calibrated, but it required data of organ functions three days after intubation [21]. Villar et al. developed a risk model categorizing continuous variables into tertiles [15]. However, tertiles may not be appropriate for some variables have intricate dependencies and associations with outcome. In the study, based on a relatively large sample size, we incorporated demographic, clinical, and laboratory variables that were available in clinical use and all collected at the admission, allowing for early recognition of ARDS patients at a high risk of death. After univariate and multivariate logistic regressions, eight predictors were finally included in the model. The model was well discriminated as reflected by an AUC of 0.791 in the training set and 0.780 in the testing set and as confirmed by the Hosmer–Lemeshow test and the calibration curve. Also, we performed an external validation using data from a Chinese hospital, and the results indicated the good predictive ability of the model in Chinese patients. In addition, we plotted a nomogram for visualizing the model, which was more convenient for clinicians to predict the mortality risk of individual patients.

Several limitations should be considered in the study. First of all, data in our study were collected from the MIMIC-III Database and our hospital. To keep the uniformity of the variables in the datasets, the selection of variables was limited in some way. Also, the accuracy and the specificity were relatively poor and the sample size in the external validation set was relatively small. In the future, a prospective study with a larger sample size is preferred for validating our model.

## 5. Conclusion

In the present study, a nomogram for predicting the risk of death in ARDS patients was developed and validated. The model incorporated eight predictors that were available in clinical use. It may help clinicians early identify ARDS patients with high risk of death, which could make timely treatment therapies and interventions for reducing the mortality and improving the survival of ARDS patients.

## Figures and Tables

**Figure 1:** The nomogram for predicting the mortality risk of ARDS.

**Figure 2:** An example for the application of the nomogram.

**Figure 3:** ROC curves and calibration curves of the training group, testing group, and validation group. (a) ROC curve of training. (b) ROC curve of testing. (c) ROC curve of validation. (d) Calibration curve of training. (e) Calibration curve of testing. (f) Calibration curve of validation.

**Table 1:** Multiple imputation and sensitivity analysis of missing data.

Variable	Missing proportion (%)	Before imputation	After imputation	Statistical	*P*
Sex	0.0				
Age	0.0				
Pathogenesis	0.0				
Respiratory rate	0.0				
Heart rate	0.0				
FIO_2_	0.0				
Heart failure	0.0				
Renal failure	0.0				
SAPS II score	0.0				
SOFA score	0.0				
Bicarbonate input	0.0				
Ventilation	0.0				
Vital status	0.0				
Survival time	0.0				
ICU type	0.0				
Immune function impairment	0.0				
Creatinine	0.0				
TBIL	24.1	0.60 (0.40, 1.20)	0.70 (0.40, 1.60)	*Z* = 1.608	0.150
AST	23.6	45.00 (28.00, 98.00)	47.00 (27.00, 109.00)	*Z* = 1.104	0.270
ALT	23.4	31.00 (18.00, 80.00)	30.00 (18.00, 76.00)	*Z* = −0.394	0.694
SaO_2_	20.0	88.25 ± 14.01	87.95 ± 13.99	*t* = 0.560	0.575
PaO_2_	20.3	169.00 (97.00, 292.00)	156.00 (93.00, 281.00)	*Z* = −1.572	0.089
Lactate	17.9	1.90 (1.30, 3.10)	2.00 (1.30, 3.20)	*Z* = 1.340	0.180
INR	0.8	1.30 (1.10, 1.60)	1.30 (1.10, 1.60)	*Z* = 0.213	0.831
Ventilation time	0.8	7.00 (3.00, 13.00)	7.00 (3.00, 14.00)	*Z* = 0.824	0.410
pH	0.3	7.34 ± 0.12	7.34 ± 0.12	*t* = 0.220	0.824
MAP	0.2	84.40 ± 17.29	84.55 ± 17.28	*t* = −0.270	0.784
GCS score	0.2	9.00 (5.00, 13.00)	9.00 (5.00, 13.00)	*Z* = −0.290	0.772
Potassium	0.2	4.24 ± 0.80	4.24 ± 0.80	*t* = −0.080	0.937
SBP	0.1	125.00 ± 26.30	124.99 ± 26.28	*t* = 0.010	0.994
Sodium	0.1	138.85 ± 4.80	138.83 ± 4.79	*t* = 0.080	0.937
RBC	0.1	3.68 ± 0.74	3.68 ± 0.74	*t* = −0.070	0.945
Hemoglobin	0.1	11.09 ± 2.18	11.09 ± 2.18	*t* = −0.060	0.956
WBC	0.1	12.70 (9.20, 17.30)	12.70 (9.20, 17.40)	*Z* = 0.032	0.975
Bicarbonate	0.1	23.35 ± 4.71	23.35 ± 4.70	*t* = 0.020	0.988
Hematocrit	0.1	32.89 ± 6.32	32.90 ± 6.32	*t* = −0.040	0.971
PLT	0.1	219.00 (153.00, 301.00)	219.00 (153.00, 301.00)	*Z* = −0.015	0.988
BUN	0.1	19.00 (14.00, 30.00)	19.00 (14.00, 30.00)	*Z* = 0.013	0.990

*Note*. SAPS II: Simplified Acute Physiology Score II; SOFA score: Sequential Organ Failure Assessment score; ICU: intensive care unit; TBIL: total bilirubin; AST: aspartate transaminase; ALT: alanine transaminase; INR: international normalized ratio; MAP: mean arterial pressure; GCS: Glasgow Coma Scale; RBC: red blood cell; WBC: white blood cell; PLT: platelet; BUN: blood urea nitrogen.

**Table 2:** Baseline characteristics of included patients.

Variable, *n* (%)	Chinese patients (*n* = 168)	MIMIC-III Database (*n* = 1814)			Statistical	*P*
		Total (*n* = 1814)	Training group (*n* = 1230)	Testing group (*n* = 584)		
*Demographic data*						
Age, years, mean ± SD	61.43 ± 17.66	62.16 ± 16.93	61.92 ± 17.31	62.66 ± 16.08	*t* = −0.890	0.375
Sex					*χ* ^2^ = 1.164	0.281
Male	100 (59.52)	1048 (57.77)	700 (56.91)	348 (59.59)		
Female	68 (40.48)	766 (42.23)	530 (43.09)	236 (40.41)		
*Laboratory indicators*						
SaO_2_, mean ± SD	90.02 ± 12.02	87.90 ± 13.99	87.88 ± 14.06	87.95 ± 13.85	*t* = −0.090	0.926
PaO_2_/FiO_2_, *M* (Q1, Q3)	29.10 (18.73, 42.30)	28.34 (16.94, 43.30)	27.31 (16.52, 42.84)	29.70 (17.94, 43.90)	*Z* = 1.922	0.056
PLT, 109/L, *M* (Q1, Q3)	220.00 (148.00, 300.00)	211.00 (145.00, 293.00)	209.00 (145.00, 288.00)	218.00 (144.50, 308.00)	*Z* = 1.250	0.211
pH, mean ± SD	7.35 ± 0.11	7.34 ± 0.12	7.34 ± 0.12	7.35 ± 0.11	*t* = −1.080	0.279
Lactate, mmol/L, *M* (Q1, Q3)	1.90 (1.35, 3.15)	2.00 (1.30, 3.20)	2.00 (1.30, 3.30)	2.00 (1.30, 3.00)	*Z* = −1.162	0.245
INR, %, *M* (Q1, Q3)	1.30 (1.10, 1.50)	1.30 (1.10, 1.50)	1.30 (1.10, 1.50)	1.30 (1.10, 1.54)	*Z* = 1.022	0.307
Creatinine, mg/dl, *M* (Q1, Q3)	1.00 (0.70, 1.30)	1.00 (0.70, 1.40)	1.00 (0.70, 1.40)	1.00 (0.70, 1.40)	*Z* = −0.417	0.677
Hematocrit, %, mean ± SD	32.66 ± 6.74	33.06 ± 6.42	33.04 ± 6.28	33.09 ± 6.71	*t* = −0.140	0.886
Hemoglobin, g/dl, mean ± SD	11.08 ± 2.31	11.11 ± 2.19	11.13 ± 2.15	11.09 ± 2.27	*t* = 0.350	0.723
AST, U/L, *M* (Q1, Q3)	57.00 (28.50, 113.00)	45.00 (28.00, 98.00)	44.00 (28.00, 98.00)	48.00 (28.00, 98.00)	*Z* = 0.427	0.669
ALT, U/L, *M* (Q1, Q3)	29.00 (17.00, 92.00)	31.00 (18.00, 75.00)	31.00 (18.00, 72.00)	34.00 (18.00, 80.00)	*Z* = 0.996	0.319
TBIL, umol/L					*χ* ^2^ = 0.068	0.794
Normal	100 (59.52)	1101 (60.69)	744 (60.49)	357 (61.13)		
Abnormal	68 (40.48)	713 (39.31)	486 (39.51)	227 (38.87)		
BUN, mg/dl					*χ* ^2^ = 1.019	0.313
Normal	146 (86.90)	1524 (84.01)	1026 (83.41)	498 (85.27)		
Abnormal	22 (13.10)	290 (15.99)	204 (16.59)	86 (14.73)		
WBC, 109/L					*χ* ^2^ = 0.009	0.925
Normal	138 (82.14)	1523 (83.96)	1032 (83.90)	491 (84.08)		
Abnormal	30 (17.86)	291 (16.04)	198 (16.10)	93 (15.92)		
Potassium, mmol/L					*χ* ^2^ = 0.358	0.550
Normal	148 (88.10)	1524 (84.01)	1029 (83.66)	495 (84.76)		
Abnormal	20 (11.90)	290 (15.99)	201 (16.34)	89 (15.24)		
Sodium, mmol/L					*χ* ^2^ = 0.052	0.820
Normal	153 (91.07)	1638 (90.30)	1112 (90.41)	526 (90.07)		
Abnormal	15 (8.93)	176 (9.70)	118 (9.59)	58 (9.93)		
Bicarbonate, mmol/L					*χ* ^2^ = 0.057	0.811
Normal	136 (80.95)	1479 (81.53)	1001 (81.38)	478 (81.85)		
Abnormal	32 (19.05)	335 (18.47)	229 (18.62)	106 (18.15)		
MAP, mean ± SD	84.89 ± 17.78	84.58 ± 17.59	84.74 ± 17.32	84.24 ± 18.15	*t* = 0.570	0.567
*Clinical data*						
ICU type					*χ* ^2^ = 2.087	0.149
Medical ICU	53 (31.55)	604 (33.30)	396 (32.20)	208 (35.62)		
Others	115 (68.45)	1210 (66.70)	834 (67.80)	376 (64.38)		
ARDS causes					*χ* ^2^ = 4.720	0.094
Pneumonia	7 (4.17)	150 (8.27)	109 (8.86)	41 (7.02)		
Sepsis	2 (1.19)	51 (2.81)	40 (3.25)	11 (1.88)		
Others	159 (94.64)	1613 (88.92)	1081 (87.89)	532 (91.10)		
Bicarbonate input					*χ* ^2^ = 1.614	0.204
No	152 (90.48)	1560 (86.00)	1049 (85.28)	511 (87.50)		
Yes	16 (9.52)	254 (14.00)	181 (14.72)	73 (12.50)		
Ventilation					*χ* ^2^ = 0.997	0.318
No	21 (12.50)	264 (14.55)	172 (13.98)	92 (15.75)		
Yes	147 (87.50)	1550 (85.45)	1058 (86.02)	492 (84.25)		
Ventilation time, days, *M* (Q1, Q3)	7.00 (2.50, 14.00)	7.00 (3.00, 15.00)	8.00 (3.00, 15.00)	7.00 (3.00, 15.00)	*Z* = −0.731	0.465
SAPS II, *M* (Q1, Q3)	36.00 (29.00, 47.00)	38.00 (29.00, 48.00)	38.00 (29.00, 48.00)	39.00 (29.00, 47.50)	*Z* = 0.263	0.793
GCS score, *M* (Q1, Q3)	9.00 (5.00, 13.00)	9.00 (5.00, 14.00)	8.00 (4.00, 13.00)	9.00 (5.00, 14.00)	*Z* = 1.736	0.068
SOFA score, *M* (Q1, Q3)	6.00 (4.00, 9.00)	6.00 (4.00, 9.00)	7.00 (4.00, 9.00)	6.00 (4.00, 9.00)	*Z* = −0.453	0.650
Immune function impairment					*χ* ^2^ = 0.567	0.452
No	127 (75.60)	1270 (70.01)	868 (70.57)	402 (68.84)		
Yes	41 (24.40)	544 (29.99)	362 (29.43)	182 (31.16)		
Heart failure					*χ* ^2^ = 0.294	0.588
No	116 (69.05)	1261 (69.51)	860 (69.92)	401 (68.66)		
Yes	52 (30.95)	553 (30.49)	370 (30.08)	183 (31.34)		
Renal failure					*χ* ^2^ = 0.001	0.975
No	113 (67.26)	1203 (66.32)	816 (66.34)	387 (66.27)		
Yes	55 (32.74)	611 (33.68)	414 (33.66)	197 (33.73)		
Respiratory rate, breaths/min, *M* (Q1, Q3)	16.00 (14.00, 23.00)	18.00 (14.00, 24.00)	19.00 (14.00, 24.00)	18.00 (14.00, 24.00)	*Z* = −1.214	0.225
Heart rate, breaths/min, mean ± SD	91.51 ± 21.17	94.13 ± 21.11	94.36 ± 21.49	93.64 ± 20.30	*t* = 0.670	0.500
Outcome					*χ* ^2^ = 1.165	0.280
Survival	90 (53.57)	942 (51.93)	628 (51.06)	314 (53.77)		
Death	78 (46.43)	872 (48.07)	602 (48.94)	270 (46.23)		

*Note*. ICU: intensive care unit; ARDS: acute respiratory distress syndrome; AST: aspartate transaminase; ALT: alanine transaminase; INR: international normalized ratio; RBC: red blood cell; PLT: platelet; TBIL: total bilirubin; BUN: blood urea nitrogen; WBC: white blood cell; MAP: mean arterial pressure; SAPS II: Simplified Acute Physiology Score II; GCS: Glasgow Coma Scale; SOFA score: Sequential Organ Failure Assessment score.

**Table 3:** Univariate logistic analysis of the training group.

Variable, *n* (%)	Training group (*n* = 1230)	Outcome		Statistical	*P*
		Survival (*n* = 628)	Death (*n* = 602)		
Age, years, mean ± SD	61.92 ± 17.31	55.30 ± 17.78	68.83 ± 13.77	*t* = −14.970	<0.001
Sex				*χ* ^2^ = 0.172	0.678
Male	700 (56.91)	361 (57.48)	339 (56.31)		
Female	530 (43.09)	267 (42.52)	263 (43.69)		
SaO_2_, mean ± SD	87.88 ± 14.06	88.34 ± 13.13	87.41 ± 14.97	*t* = 1.160	0.246
PaO_2_/FiO_2_, *M* (Q1, Q3)	27.31 (16.52, 42.84)	30.46 (18.17, 46.58)	24.54 (15.00, 37.62)	*Z* = −5.321	<0.001
PLT, *M* (Q1, Q3)	209.00 (145.00, 288.00)	207.50 (149.00, 281.00)	210.00 (137.00, 293.00)	*Z* = 0.162	0.871
pH, mean ± SD	7.34 ± 0.12	7.34 ± 0.12	7.34 ± 0.12	*t* = 0.260	0.795
Lactate, *M* (Q1, Q3)	2.00 (1.30, 3.30)	1.90 (1.30, 3.30)	2.00 (1.40, 3.30)	*Z* = 1.014	0.311
INR, *M* (Q1, Q3)	1.30 (1.10, 1.50)	1.20 (1.10, 1.40)	1.30 (1.20, 1.70)	*Z* = 6.092	<0.001
Creatinine, *M* (Q1, Q3)	1.00 (0.70, 1.40)	0.90 (0.70, 1.20)	1.10 (0.80, 1.60)	*Z* = 5.050	<0.001
Hematocrit, mean ± SD	33.04 ± 6.28	33.64 ± 6.47	32.42 ± 6.02	*t* = 3.440	<0.001
Hemoglobin, mean ± SD	11.13 ± 2.15	11.39 ± 2.24	10.85 ± 2.02	*t* = 4.470	<0.001
AST, *M* (Q1, Q3)	44.00 (28.00, 98.00)	45.00 (29.00, 95.00)	43.00 (27.00, 104.00)	*Z* = −0.455	0.649
ALT, *M* (Q1, Q3)	31.00 (18.00, 72.00)	30.00 (19.00, 64.00)	31.00 (17.00, 88.00)	*Z* = 0.844	0.399
TBIL				*χ* ^2^ = 14.059	<0.001
Normal	744 (60.49)	412 (65.61)	332 (55.15)		
Abnormal	486 (39.51)	216 (34.39)	270 (44.85)		
BUN				*χ* ^2^ = 26.937	<0.001
Normal	1026 (83.41)	490 (78.03)	536 (89.04)		
Abnormal	204 (16.59)	138 (21.97)	66 (10.96)		
WBC				*χ* ^2^ = 0.088	0.767
Normal	1032 (83.90)	525 (83.60)	507 (84.22)		
Abnormal	198 (16.10)	103 (16.40)	95 (15.78)		
Potassium				*χ* ^2^ = 3.793	0.051
Normal	1029 (83.66)	538 (85.67)	491 (81.56)		
Abnormal	201 (16.34)	90 (14.33)	111 (18.44)		
Sodium				*χ* ^2^ = 0.021	0.884
Normal	1112 (90.41)	567 (90.29)	545 (90.53)		
Abnormal	118 (9.59)	61 (9.71)	57 (9.47)		
Bicarbonate				*χ* ^2^ = 1.028	0.311
Normal	1001 (81.38)	518 (82.48)	483 (80.23)		
Abnormal	229 (18.62)	110 (17.52)	119 (19.77)		
MAP, mean ± SD	84.74 ± 17.32	86.06 ± 17.74	83.38 ± 16.77	*t* = 2.720	0.007
ICU type				*χ* ^2^ = 1.743	0.187
Medical ICU	834 (67.80)	415 (66.08)	419 (69.60)		
Others	396 (32.20)	213 (33.92)	183 (30.40)		
ARDS cause				*χ* ^2^ = 2.190	0.334
Pneumonia	109 (8.86)	56 (8.92)	53 (8.80)		
Sepsis	40 (3.25)	25 (3.98)	15 (2.49)		
Others	1081 (87.89)	547 (87.10)	534 (88.70)		
Bicarbonate input				*χ* ^2^ = 9.770	0.002
No	1049 (85.28)	555 (88.38)	494 (82.06)		
Yes	181 (14.72)	73 (11.62)	108 (17.94)		
Ventilation				*χ* ^2^ = 33.480	<0.001
No	1058 (86.02)	505 (80.41)	553 (91.86)		
Yes	172 (13.98)	123 (19.59)	49 (8.14)		
Ventilation time, *M* (Q1, Q3)	8.00 (3.00, 15.00)	8.00 (3.00, 15.00)	7.00 (3.00, 15.00)	*Z* = 0.183	0.855
SAPS II, *M* (Q1, Q3)	38.00 (29.00, 48.00)	32.50 (21.00, 41.00)	43.00 (35.00, 53.00)	*Z* = 13.604	<0.001
GCS score, *M* (Q1, Q3)	8.00 (4.00, 13.00)	8.00 (3.00, 13.00)	9.00 (5.00, 13.00)	*Z* = 1.529	0.126
SOFA score, *M* (Q1, Q3)	7.00 (4.00, 9.00)	6.00 (3.00, 8.00)	7.00 (5.00, 10.00)	*Z* = 6.820	<0.001
Immune function impairment				*χ* ^2^ = 30.088	<0.001
No	868 (70.57)	487 (77.55)	381 (63.29)		
Yes	362 (29.43)	141 (22.45)	221 (36.71)		
Heart failure				*χ* ^2^ = 69.255	<0.001
No	860 (69.92)	506 (80.57)	354 (58.80)		
Yes	370 (30.08)	122 (19.43)	248 (41.20)		
Renal failure				*χ* ^2^ = 76.323	<0.001
No	816 (66.34)	489 (77.87)	327 (54.32)		
Yes	414 (33.66)	139 (22.13)	275 (45.68)		
Respiratory rate, *M* (Q1, Q3)	19.00 (14.00, 24.00)	19.00 (14.00, 24.00)	18.00 (14.00, 24.00)	*Z* = −1.590	0.112
Heart rate, mean ± SD	94.36 ± 21.49	95.36 ± 21.12	93.32 ± 21.83	*t* = 1.660	0.097

*Note*. ICU: intensive care unit; ARDS: acute respiratory distress syndrome; AST: aspartate transaminase; ALT: alanine transaminase; INR: international normalized ratio; RBC: red blood cell; PLT: platelet; TBIL: total bilirubin; BUN: blood urea nitrogen; WBC: white blood cell; MAP: mean arterial pressure; SAPS II: Simplified Acute Physiology Score II; GCS: Glasgow Coma Scale; SOFA score: Sequential Organ Failure Assessment score.

**Table 4:** Multivariate logistic analysis of the training group.

Variable	*β*	S.E.	Wald	*P*	OR	95% CI	
						Lower	Upper
Constant	−3.147	0.503	39.089	<0.001			
Age	0.037	0.005	60.606	<0.001	1.037	1.028	1.047
Hemoglobin	−0.068	0.032	4.527	0.033	0.934	0.877	0.995
Heart failure (yes)	0.522	0.149	12.254	<0.001	1.686	1.258	2.258
Renal failure (yes)	0.487	0.148	10.778	0.001	1.628	1.217	2.178
SAPS II	0.029	0.005	36.141	<0.001	1.029	1.020	1.039
Immune function impairment (yes)	0.697	0.149	21.800	<0.001	2.007	1.498	2.689
TBIL (abnormal)	0.279	0.136	4.209	0.040	1.322	1.013	1.727
PaO_2_/FiO_2_	−0.006	0.003	4.635	0.031	0.995	0.990	0.999

*Note*. S.E.: standard error; OR: odds ratio; CI: confidence interval; SAPS II: Simplified Acute Physiology Score II; TBIL: total bilirubin.

**Table 5:** Assessment and validation of the prediction model.

Parameter	Dataset		
	Training group	Testing group	External validation
AUC (95% CI)	0.791 (0.766–0.816)	0.780 (0.743–0.816)	0.758 (0.756–0.761)
Accuracy (95% CI)	0.730 (0.705–0.755)	0.697 (0.660–0.734)	0.696 (0.627–0.766)
Sensitivity (95% CI)	0.822 (0.792–0.853)	0.804 (0.756–0.851)	0.756 (0.661–0.852)
Specificity (95% CI)	0.642 (0.604–0.679)	0.605 (0.551–0.659)	0.644 (0.546–0.743)

*Note*. AUC: area under the curve; CI: confidence interval.

## Data Availability

The data used to support the findings of this study are available from the corresponding author upon request.
